# 3D CNN with Visual Insights for Early Detection of Lung Cancer Using Gradient-Weighted Class Activation

**DOI:** 10.1155/2021/6695518

**Published:** 2021-03-11

**Authors:** Eali Stephen Neal Joshua, Debnath Bhattacharyya, Midhun Chakkravarthy, Yung-Cheol Byun

**Affiliations:** ^1^Department of Computer Science and Multimedia, Lincoln University College, Kuala Lumpur 47301, Malaysia; ^2^Department of Computer Science and Engineering, Koneru Lakshmaiah Education Foundation, K.L. University, Guntur 522502, Andhra-Pradesh, India; ^3^IIST, Department of Computer Engineering, Jeju National University, Jeju 63243, Republic of Korea

## Abstract

The 3D convolutional neural network is able to make use of the full nonlinear 3D context information of lung nodule detection from the DICOM (Digital Imaging and Communications in Medicine) images, and the Gradient Class Activation has shown to be useful for tailoring classification tasks and localization interpretation for fine-grained features and visual explanation for the internal working. Gradient-weighted class activation plays a crucial role for clinicians and radiologists in terms of trusting and adopting the model. Practitioners not only rely on a model that can provide high precision but also really want to gain the respect of radiologists. So, in this paper, we explored the lung nodule classification using the improvised 3D AlexNet with lightweight architecture. Our network employed the full nature of the multiview network strategy. We have conducted the binary classification (benign and malignant) on computed tomography (CT) images from the LUNA 16 database conglomerate and database image resource initiative. The results obtained are through the 10-fold cross-validation. Experimental results have shown that the proposed lightweight architecture achieved a superior classification accuracy of 97.17% on LUNA 16 dataset when compared with existing classification algorithms and low-dose CT scan images as well.

## 1. Introduction

Lung cancer is the most commonly [1] discovered dangerous cells and additionally one of the most perilous cancer tissues that lead to fatality among males in 2019. Exactly, bronchi cancer tissues have actually happened to be a primary risk to personal everyday lifestyle. Low-dose computed tomography (CT) is actually a valuable method for pinpointing lung cancer tissues [2] early. A choice to recognition through these predefined features is by using component finding methods to find first-class depictions straight from the instruction [3] and relevant information. Convolutional neural networks (CNNs), like a swiftly, scalable, and also end-to-end finding-out neural network, considerably evolved the landscape of goal findings, such as in image classification, medical diagnosis [4], and semantic division.

Thoracic CT creates a volume of pieces that may be regulated to reveal several volumetric pictures of physical structures in the bronchi. 2D convolution dismisses the 3D spatial size, indicating that it is actually incapable of making complete usage of the 3D condition pertinent [5] information, and 3D CNN can, definitely, be in harmony with this. Our goal is to check empirically the trouble of determining bronchi acnes captured through computed tomography (CT) in an end-to-end means making usage of the 3D convolutional neural network (CNN) effectively to perform a binary distinction [6] (benign and malignant) on CT pictures [7] from the Lung Image Database Consortium picture variety (LUNA 16 Dataset). Our major contributions are as follows:

1. 3D CNN is used for the automated distinction of bronchi blemishes. Reviewed with the 2D design, 3D CNNs can effortlessly encode richer spatial information to eliminate additional unique symbols.
2. Multiview places are actually utilized in our designs. Our staff use the multiview-one-network strategy that contrasts and arises from the one-view-one-network technique used in the study. Completion leads to the fact that our technique may achieve a decreased mistake rate than the one-view-one-network approach while using far fewer requirements. Note that while the layout used a similar approach and 2D CNN is simply utilized, our group used 3D CNN in this paper.
3. To the best of our knowledge, this is the first study to use 3D AlexNet substitutes of Inception as well as Inception-ResNet to categorize lung imperfections.
4. Our model attained a much better outcome than the remaining models associated with the differences in CT.

We utilize 3D CNN for the automatic distinction of lung Cancer. The 2D multiview areas are actually used in our styles. Our team used the improvised 3D AlexNet.

Recently, deep neural nets have shown superior performance and classification problems and 2D convolutional neural networks [8]; they look at a slice of the CT scan normally. CT scan data is 3D [9], so it will have many different slices. 2D CNN scans multiple angles [10] of that CT scan data and then that can allow for higher accuracy. So, obviously, 2D CNN is one approach but 3D CNN uses the full nature of the 3D data. Instead of the 2D data, we are having higher accuracy and specifically low knowledge section tasks, and we can think about this from the human perspective to get a better idea. This allows them to do a better diagnosis [11] of whether it is a lung nodule or not, so the same thing applies to the convolutional neural network.

This paper is organized as follows. In Section 2, related work and gap identification were thoroughly reviewed.  Section 3 deals with the overview 2D convolutional neural network and 3D CNN and utilization for the current problem.  Section 4 proposed the work, and Section 5 explains the experimental results and analysis.

## 2. Related Works

Lung cancer is the leading cause of cancer deaths for both men and women, making up almost 26% of all cancer deaths worldwide. The survival rate for five years is just 17 percent. Early diagnosis increases the probability of success and prognosis dramatically. Owing to the amount of data involved, diagnosis of lung nodules is time-intensive and often suffers from interradiology heterogeneity. A commonly used method for screening for lung cancer is computed tomography (CT). The purpose of screening is to diagnose infection at the earliest possible point.

In [12], LIDC/IDRI dataset is used where the researchers have used the intrinsic CNN features, and 431 malignant nodules and 795 benign nodules were extracted, and the input for SVM was sequential forward feature method to construct the classifier. The researchers attained an accuracy of 85%.

In [13], LUNA 16 dataset is used where the researchers proposed the deep hierarchical semantic convolutional neural network with cross-validation and achieved an accuracy of 89%; 1386 nodules were used: 90% is for testing and 10% is for training.

In [14], LUNA 16 dataset is used where researchers performed a two-stage convolutional neural network strategy. The first stage is to refine the input CT image, and the second stage is simplified Google Nets for improvised classification. The authors have achieved an accuracy of 89.6% where they used 90% for training and 10% for testing out of 888 thoracic cancer images. In [15], LUNA 16 dataset is used where the researchers used 11 Deep CNN models. Modified CNN architecture integrated them and adopted transfer learning. An accuracy of 88% was achieved (0.94).

In [16], LUNA 16 dataset was investigated with 3D convolutional neural network techniques. Researchers tried to reduce the false-positive ratio in the first stage and used the classification label over union self-normalization and interclass variation for density, shape, and size. They achieved an accuracy of 91% with 888 thoracic images with 90% for testing and 10% for training. The 3D convolutional neural network was used for differentiating preinvasive lesions from invasive adenocarcinomas appearing on ground glass nodules with diameter <3 cm using HRCT'. In [17], LUNA 16 dataset was used. The authors adopted a 3N convolutional neural network and processed using the lung mask extraction and achieved an accuracy of 89%.

In [18], the UCI dataset is used as an input and the authors used binarization procedure to contrast it with edges to identify the lung cancer growth. The researchers [19] had used multiview convolutional neural network and conducted binary classification and ternary classification. They achieved an accuracy of 70.7% on the LIDC-IDRI dataset. The authors stated that by using multiview convolutional neural network, the error rate can be decreased. Soft activation mapping [20] techniques were used for finding the low-grade malignant nodule. For feature selection, the authors used a high-level feature enhancement scheme to localize the shape nodule. The researchers in [21] used the pretrained weighted model on the LIDC-IDRI dataset and feature selection and handcrafted texture descriptors and achieved an accuracy of 78%. The literature survey from [12–18] clearly shows that classification of the lung nodule should be improvised with better accuracy, and in [19–21], the authors had proposed a heavyweight model due to which the training process takes an enormous amount of time, and also it will give different results on different machines. It is not interpretable to individuals in the domain, no matter how strong the deep learning model is. It is very difficult for them to follow it. So, all models have recently been known to have very strong accuracies, particularly deep learning models. But if the domain specialist does not believe the model, it does not mean much. Since it will not really gain acceptance, the idea is how we can use techniques such as gradient-weighted class activation mapping or Grad-CAM to visualize the decision-making of the model and increase the trust of radiologists and enhance adoption in the field by employing the lightweight process model.

## 3. Convolutional Neural Network

A new architecture called a convolutional neural network (CNN) [22] consists of the input and output like any other deep learning method and it will have layers called convolutional layers and max-pooling layers. The general idea summary is shown in Figure 1.

The general idea is that the input will go through a series of convolution and max-pooling layers, just like other researchers [23], and then this will map some fully connected layers at the end which map an output.

### 3.1. Convolutional Layer

The kernel will convolve [24] over the input, so it will start at the left and will go to the next layer, and then dot product is taken between the kernel and the input. This output feature map like convolution neural layers can detect certain features in the image.  Figure 2 explains the working of 2D Kernal and the sliding of Kernal over the input image. The feature was extracted from the convolution layer.

### 3.2. Max-Pooling Layers

The idea is that convolution layers can detect the edges of the little edges on the CT scan. The convolutional layers can detect certain parts of the CT scan which may be the benign nodule or the malignant nodule, and finally, the last few layers will detect the entire benign nodule.  Figure 3 shows a 3D kernel for the proposed architecture. So, this is the main layer that makes up the convolutional neural network.

But another critical layer is also the max-pooling layers which basically take the max value in a certain area and pull it into a singular value. Max pooling is actually a merging procedure that decides on the maximum component coming from the area of the attribute chart dealt with due to the filter. Hence, the outcome after max-pooling level would certainly be a feature chart having the most prominent highlights of the previous feature map. The max-pooling layer reduces the dimensions [25] of the data and this allows for quicker computation.

Max-pooling layers which reduce dimensions allow for better computational speed and reduce overfitting. So, each CNN layer has features of increasing complexity. The first layer learns edges and corners things like that, and then, as we go further, the intermediate layers will learn more complex parts of the object, and finally, the last layers will detect full objects.

### 3.3. 3D Convolutional Neural Network

3D CNN is essentially the same thing except for the fact that your input will be 3D data, instead of being a singular layer. Filters will also be 3D. So instead of detecting 2D features such as edges and corners, it will detect the same features but in the 3D fashion [26], which is really critical especially in this lung nodule case because all the data is of 3D nature.

The working idea is that this 3D data is inputted. It goes through some 3D kernels and then it is classified as either healthy or diseased; in this case, one module exists in that CT image or a long module does not exist. So, in addition to this CNN, other deep neural network medical image analyses [27] have been black boxes giving users no intuition as to how they are predicting.  Figure 4 shows the architecture of 3D CNN.

## 4. Proposed Model

The superior outcome in real-time environments is not proven to be effective; however, due to the lack of transparency in the previous models, there are esteem challenges for real-life implementation. By highlighting discriminative areas, gradient-weighted class activation mapping (Grad-CAM) offers visual descriptions. This research produces a 3D CNN for better confidence and acceptance with state-of-the-art precision and visual perspectives. In the process of debugging and optimization, visual perspectives help. The first study reveals that in lung nodule classification, Grad-CAM techniques [28] will provide visual interpretations for model decisions. 3D convolution neural networks that make good use of the 3D structure of input data detect lung nodules with greater precision. The flow of the suggested architecture is shown in Figure 5.

### 4.1. Gradient Weight Class Activation

Gradient-weighted class activation mapping techniques can provide visual explanations for model decisions in lung nodule detection by highlighting discriminative regions. This is a very powerful approach for figuring out how we can make the model interpretable for people in the domain. We provide visual insights into how exactly the model is making its decision. This will allow for better trust and adoption in the field, in addition to validating the model and updating it across the debugging and optimization process. We can look at these visual insights and see where the model is failing and why the model is failing, and we can address this by changing the architecture of the model. This study demonstrates Grad-CAM techniques for visual nations on one module classification. The objective here is to research and develop 3D CNN to detect lung nodules and CT scan data with better accuracy and higher trust in existing models, and this is to ultimately aid in the early detection of lung cancer to improve chances of survival and prognosis.

(1) $$\begin{array}{c} Y_{\text{Grad}-\text{Cam}}^{a}=\sum_{p}^{1}w_{p}^{q}\frac{1}{z}\sum_{i}1\sum_{j}A_{ij}^{p}. \end{array}$$

Let us define *J*^*p*^ to be average pooled global output.

(2) $$\begin{array}{c} J^{p}=\frac{1}{z}\sum_{i}*\sum_{j}A_{ij}^{p}. \end{array}$$

Grad-CAM computes the end scores by

(3) $$\begin{array}{c} Y_{\text{Grad}-\text{Cam}}^{a}=\sum_{p}^{1}*w_{p}^{q}*J^{p}, \end{array}$$

where *w*_*p*_^*q*^ is the weight connecting the Kth Feature map.

Taking the gradient class score (*J*^*p*^) w.r.t to feature map, we get

(4) $$\begin{array}{c} \frac{\delta y_{1}^{c}}{\delta J_{1}^{p}}=\frac{\delta y^{c}/\delta A_{ij}^{p}}{\delta J^{p}/\delta A_{ij}^{p}}. \end{array}$$

Taking partial derivation (4) w.r.t. *A*_*ij*_^*p*^, we can see that *δJ*^*p*^/*δA*_*ij*_^*p*^ = 1/*z*. Substituting this into (4), we get

(5) $$\begin{array}{c} \frac{\delta y_{1}^{c}}{\delta J_{1}^{p}}=\frac{\delta y^{c}}{\delta A_{ij}^{p}}*z. \end{array}$$

From (3), we get

(6) $$\begin{array}{c} w_{p}^{q}=z*\frac{\delta J^{p}}{\delta A_{ij}^{p}}. \end{array}$$

Summing both sides of (6),

(7) $$\begin{array}{c} \sum_{i}\sum_{j}W_{p}^{q}=\sum_{i}\sum_{j}z*\frac{\delta y^{c}}{\delta A_{ij}^{p}}. \end{array}$$

Therefore,

(8) $$\begin{array}{c} w_{p}^{q}=\sum_{i}\sum_{j}\frac{\delta y^{c}}{\delta A_{ij}^{p}}. \end{array}$$

We may thus conclude that Grad-CAM is a strict CAM generalization. This generalization helps the researcher to produce a visual description from the 3D CNN-based model for professional developers that will make the method streamlined and convoluted. As a result, in the computer tomography images, we can get the same nodule area. We execute a weighted combination of activation maps of forwarding and follow it with a ReLu to obtain the following equation for the nonlinearity. Activation function has been applied to each layer component of the output feature map; thus, due to this, it will add nonlinearity to the CNN. We have used the rectified linear unit as the activation function in the proposed algorithm. It works as follows:

(9) $$\begin{array}{c} {\text{LN}}_{\text{Grad}-\text{Cam}}^{a}=\text{ReLu}\left(\sum_{k}\alpha_{k}^{c}A^{k}\right). \end{array}$$

## 5. Experimental Results and Discussion

### 5.1. LUNA 16 Dataset

LUNA 16 dataset [29] includes 888 clinical thoracic CT scans. CT scans with slice thickness greater than 3 mm or with inconsistent slice spacing were excluded. Image annotation was done by four experienced thoracic radiologists. Each radiologist marked the lesions they identified as nonnodule, nodule <3 mm, and nodules > = 3 mm. The reference standard is all nodules > = 3 mm accepted by at least 3 out of 4 radiologists.  Figure 6 shows the benign and malignant images.

### 5.2. Study Design

We split the data into training and testing datasets as well as validation. We design and implement a model, and we train that model to validate that model on the validation dataset. And we iterate through this process to know how our model is performing. We can change the architecture, we can put on average pooling, and we can add more layers to change the filter sizes. We want to know how exactly we can make the model as good as possible and then we evaluate our test dataset, so the idea here is that the test dataset can only be used once because we do not want to train for test dataset or optimize the model for the test dataset. The idea is that we hold out a test dataset to be used at the very end only once, and finally we visualize a model using Grad-CAM.  Figure 7 shows the study design.

### 5.3. Split and Preprocess Data

A balanced dataset of 1,000 nodules and 1,000 nonnodule volumes was used. Data were divided into three sets for training, validation, and testing, randomized, and split into 1,400 volumes for training and 600 for testing. 10% of the training data (140 volumes) was used for validation.

### 5.4. Architecture and Implementation

From the tables, we will summarize various architecture models.  Table 1 explains the AlexNet 2D (H. Xie et al., 2019) [3], Table 2 explains the AlexNet 3D (IEEE Signal Processing Society, n.d.) [16] model, and Table 3 summarizes the proposed architecture network model. In our improvised algorithm, the network size used was 27 : 27 : 27 : 16, and we have chosen random weight max values as 1. The generalization behavior of our network with various obtained results was fixed size but the network training size was increasing.

### 5.5. Training Process

Figure 8 explains the training process on the LUNA 16 dataset. Images *X* from the training dataset were fed into the model. The output was compared with the training label *y*, the loss is computed, and the model is updated with new parameters. During the iterative training process, a SoftMax activation function was used on the estimates before the loss was calculated. Cross-entropy was used as the loss function to be optimized. All the models used Adam optimizer with a learning rate of 0.0001 and default parameters *β*1 = 0.9 and *β*2 = 0.999.  Table 4 explains the key matrices.

## 6. Results and Discussion

The “Area Under Curve” (AUC) is revealed once we make a distinction between the binary classification effectiveness and that of additional classifiers. The curve explains the receiver operating characteristic (ROC), a normal strategy for concise classifier enactment over a range of compromises among actual positive along with false-positive mistake prices. The AUC is an approved typical efficiency statistic for a ROC curve and approaches the chance that the classifier or feature will absolutely place randomly selected beneficial circumstances above arbitrarily chosen damaging circumstances. That is, the AUC can be made to represent the classifier's capability to recognize examples. High AUC numbers close to 1 indicate a good measure of separability. The proposed 3D CNN performed the best with an AUC of 97%.  Figure 9 shows the performance matrices.

Model performance key metrics and also visual insights were generated through the area elevation curve (AEC). The CNNs had good AEC close to one showing that they have a good supper ability and they are able to perform well in the detection task. Alex 3D CNN with an AEC of 95% performed better than the 2D CNN with 94%, and the proposed 3D CNN performed the best with an AUC of 97%, which shows that these optimizations that are done over iterations and validated are effective in increasing the model classification ability.

We need to highlight that this 94% recall value might only be three percent greater than Alex Net 2D CNN, but even a point zero one increase in the recall is like saving another patient living out of 100. This recall value is really critical. In particular, by maintaining the same precision, we able to increase this recall without sacrificing too much in precision. We are basically finding patients who were not suffering from cancer and found them by early detecting this long module.

The accuracy of the AlexNet of the 3D CNN is better than that of the 2D CNN. The optimized 3D CNN performed the best and it also has better recall precision values compared to the 2D CNN. So this is probably the most critical part of it as it provides visual insights into the model decision-making. Tables 5 and 6 show the performance of the proposed model in comparison to other models.

Finalized CNN was visualized using Grad-CAM to understand how the model is making decisions.

In Figure 10, the images on the left are the input images that are fed into the network. We used the images on the right for the Grad-CAM-generated maps. From the map out of a full CT scan, we can show exactly what point on that huge CT scan is giving an insight into the radiology.

The effectiveness of applying gradient-weighted class activation mapping shows how it can really provide good visual explanations to the fact that why the model is predicting what it is predicting, so this is quite critical because, sometimes, the general theme is that if you can really make the model interpretable, it can be really useful to clinicians and radiologists in terms of trusting and adopting the model, and all practitioners do not just want to have a model that can provide high accuracies but really wanted to do something in the actual field, so that is why this Grad-CAM analysis is so critical.

## 7. Conclusions

In this paper, three crucial deep neural networks were made and also widely assessed. The forecast in the classification of benign and malignant lung blemishes was contrasted in LUNA 16 dataset. The experimental outcomes suggest that the improvised 3D-CNN archived the very best efficiency than the 2D AlexNet and 3D AlexNet. The layers of the semantic network in this paper are reasonably tiny and light, because of the constraints of the data collections. The proposed approach can be expected to boost the accuracy of the other data sources. The technique can be generalized to the style of high-performance CADx systems for other medical imaging jobs in the future.

## 8. Future Work

In turn, the class activation maps are analyzed to refine the network to succeed in conditions where it does not perform well. The CNN uses max-pooling to address the problem which is class invariants, but for the biomedical images, we need class equivalence, but the major issue here is that a lot of significant data is lost in the process, and also CNN is a bad representation to the human visual system. Capsule neural network is the best and uses class equivalence to store and mimic the human vision system. Its significance indicates that capsule neural networks can train on far less data and produce more accurate results.

## Figures and Tables

**Figure 1:** Convolutional neural network.

**Figure 2:** Input and output feature maps over convolutional layer.

**Figure 3:** Max pooling in CNN.

**Figure 4:** 3D CNN architecture for lung cancer classification.

**Figure 5:** Proposed architecture.

**Figure 6:** (a) Nodule image. (b) Nonnodule image.

**Figure 7:** The study design of the proposed model for lung cancer classification.

**Figure 8:** The training process of the model.

**Figure 9:** Performance metrics of the proposed model with other models.

**Figure 10:** Visualizing the trained CNN original images on the left. Grad-CAM images on the right.

**Table 1:** AlexNet 2D CNN model.

Layer	Output shape	Param (#)
Conv 2d (conv 2D)	(None 32, 32, 16)	272
Batch_normalization_v1	(None 32, 32, 16)	64
Max_pooling 2D	(None 32, 32, 16)	0
Conv2d_1	(None 32, 32, 32)	4640
Batch_normalization_v1_1	(None 32, 32, 32)	128
Max_pooling 2d_1	(None 32, 32, 32)	0
Conv2d_2	(None 32, 32, 64)	18496
Batch_normalization_v1_2	(None 32, 32, 32)	256
Conv2d_3	(None 32, 32, 32)	36928
Batch_normalization_v1_3	(None 32, 32, 32)	256
Conv2d_4 (conv 2D)	(None 8, 8, 32)	18454
Batch_normalization_v1_4	(None 8, 8, 32)	128
Max_pooling 2d_2	(None 8, 8, 32)	0
Flatten layer	(None, 512)	0
Dense layer	(None, 200)	102600
Batch_normalization_v1_5	(None, 200)	800
Dropout (dropout)	(None, 200)	0
Dense_1 (dense layer)	(None, 75)	15075
Batch_normalization_v1_6	(None, 75)	300
Dropout_1 (dropout)	(None, 75)	0
Dense_2 (dense)	(None, 2)	152

**Table 2:** AlexNet 3D CNN model.

Layer	Output shape	Param (#)
Conv 3d_1 (conv 3D)	(None 32, 32, 32, 16)	8208
Batch_normalization_v1	(None 32, 32, 32, 16)	64
Max_pooling 3D_1	(None 16, 16, 16, 16)	0
Conv3d_1 (Conv 3D)	(None 16, 16, 16, 32)	13856
Batch_normalization_v1_2	(None 16, 16, 16, 32)	128
Max_pooling3d_2	(None 8, 8, 8, 312)	0
Conv3d_3	(None 8, 8, 8, 64)	55360
Batch_normalization_v1_3	(None 8, 8, 8, 64)	256
Conv3d_4	(None 8, 8, 8, 64)	110656
Batch_normalization_v1_4	(None 8, 8, 8, 64)	256
Conv3d_5 (conv 2D)	(None 8, 8, 8, 32)	53328
Batch_normalization_v1_5	(None 8, 8, 8, 32)	128
Max_pooling2d_3	(None 4, 4, 4, 32)	0
Falatten_1 (flatten layer)	(None, 2048)	0
Dense_1 (dense layer)	(None, 200)	409800
Batch_normalization_v1_6	(None, 200)	800
Dropout_1 (dropout)	(None, 200)	0
Dense_2 (dense layer)	(None, 75)	15075
Batch_normalization_v1_7	(None, 75)	300
Dropout_2 (dropout)	(None, 75)	0
Dense_3 (dense)	(None, 2)	152

**Table 3:** Proposed 3D CNN model.

Layer	Output shape	Param (#)
Conv 3d_1 (conv 3D)	(None 27, 27, 27, 16)	3472
Batch_normalization_v1	(None 27, 27, 27, 16)	64
Conv3d_1 (Conv 3D)	(None 27, 27, 27, 16)	2064
Batch_normalization_v1_2	(None 27, 27, 27, 16)	64
Conv3d_3	(None 27, 27, 27, 16)	16400
Max_pooling3d_2	(None 8, 8, 8, 312)	0
Batch_normalization_v1_3	(None 23, 23, 23, 16)	64
Max_pooling3d_1	(None 11, 11, 11, 16)	0
Conv3d_4	(None 10, 10, 10, 32)	4128
Batch_normalization_v1_4	(None 10, 10, 10, 32)	128
Conv3d_5 (conv 2D)	(None 9, 9, 9, 32)	8224
Batch_normalization_v1_5	(None 9, 9, 9, 32)	128
Max_pooling3d_2	(None 4, 4, 4, 32)	0
Conv3d_6 (conv 2D)	(None, 3, 3, 3, 64)	16448
Dense_1 (dense layer)	(None, 200)	409800
Batch_normalization_v1_6	(None, 3, 3, 3, 64)	256
Max_pooling3d_3	(None, 1, 1, 1, 64)	0
Flatten_1 (Flatten layer)	(None, 64)	0
Dense_1 (dense layer)	(None, 256)	16640
Batch_normalization_v1_7	(None, 256)	1024
Dropout_1 (dropout)	(None, 256)	0
Dense_2 (dense)	(None, 2)	514

**Table 4:** Key matrices with definitions.

Total population		True condition	
		Condition positive	Condition negative
Predicted condition	Predicted condition positive	True positive	False positive (type I error)
	Predicted condition negative	False negative (type II error)	True negative
		True positive rate (TPR), recall, Sensitivity = ∑true positive/∑condition positive	False-positive rate (FPR) = ∑false positive/∑condition negative
		Accuracy (ACC) = (∑true positive + ∑true negative)/∑total population	Precision = ∑true positive/∑predicted condition positive
		F1 score = 1/((1/recall + 1/precision)/2)	Specificity (SPC), selectivity = ∑true negative/∑condition negative

**Table 5:** Accuracy of CNN with different models.

CNN	AUC	Accuracy	F-score	Precision	Recall
AlexNet 2D-CNN	0.94	87.67	0.89	0.85	0.91
AlexNet 3D-CNN	0.95	89.17	0.91	0.91	0.88
Proposed 3D-CNN	0.97	97.17	0.92	0.87	0.94

**Table 6:** Comparison between the existing system and the proposed system on LUNA 16 dataset.

Experimental results								
LUNA 16 dataset information				Existing method		Proposed method		
S. No	No. of samples	Training (%)	Testing (%)	Authors	Results (%)	2D AlexNet (%)	3D AlexNet (%)	Proposed 3D AlexNet (%)
1	888	90	10	Xie et al., 2019 [3]	Accuracy 88.17	Accuracy 89.45	Accuracy 90.23	Accuracy = 97.17

2	1018	90	10	Fie li et al., 2019 [16]	Accuracy 89.67	Accuracy 88.78	Accuracy 91.13	Accuracy = 97.17

## Data Availability

The data used to support the findings of this study are available from the corresponding author upon request.

## References

[1] Balakrishnan K., Dey S., Gupta T. (2019). The impact of air pollution on deaths, disease burden, and life expectancy across the states of India: the Global Burden of Disease Study 2017. *The Lancet Planetary Health*.

[2] Agrawal A., Sheng B., Li P. (2018). Computer-assisted decision support system in pulmonary cancer detection and stage classification on CT images. *Journal of Biomedical Informatics*.

[3] Xie H., Yang D., Sun N., Chen Z., Zhang Y. (2019). Automated pulmonary nodule detection in CT images using deep convolutional neural networks. *Pattern Recognition*.

[4] Labaki W. W., Gu T., Murray S. (2019). Voxel-wise longitudinal parametric response mapping analysis of chest computed tomography in smokers. *Academic Radiology*.

[5] Ardila D., Kiraly A. P., Bharadwaj S. (2019). End-to-end lung cancer screening with three-dimensional deep learning on low-dose chest computed tomography. *Nature Medicine*.

[6] Kroenke M., Hirata K., Gafita A. (2019). Voxel-based comparison and texture analysis of 18 F-FDG and 18 F-FMISO PET of patients with head-and-neck cancer. *PLoS One*.

[7] Liao F., Liang M., Li Z., Hu X., Song S. (2019). Evaluate the malignancy of pulmonary nodules using the 3-D deep leaky noisy-OR network. *IEEE Transactions on Neural Networks and Learning Systems*.

[8] Zuo W., Zhou F., Li Z., Wang L. (2019). Multi-resolution CNN and knowledge transfer for candidate classification in lung nodule detection. *IEEE Access*.

[9] Polat H., Mehr H. D. (2019). Classification of pulmonary CT images by using hybrid 3D-deep convolutional neural network architecture. *Applied Sciences (Switzerland)*.

[10] Afshar P., Mohammadi A., Plataniotis K. N., Oikonomou A., Benali H. (2019). From handcrafted to deep-learning-based cancer radiomics: challenges and opportunities. *IEEE Signal Processing Magazine*.

[11] Liu X., Faes L., Kale A. U. (2019). A comparison of deep learning performance against health-care professionals in detecting diseases from medical imaging: a systematic review and meta-analysis. *The Lancet Digital Health*.

[12] Li S., Xu P., Li B. (2019). Predicting lung nodule malignancies by combining deep convolutional neural networks and handcrafted features. *Physics in Medicine and Biology*.

[13] Rita A., Carvalho F., Cunha A. M. (2019). Faculdade de engenharia da universidade do porto 3D lung nodule classification in computed tomography images.

[14] Yang A., Hu T., Wang J., Lyu J., Banerjee S., Ling S. H. Lung nodule classification using a novel two-stage convolutional neural networks structure.

[15] Zhao X., Qi S., Zhang B. (2019). Deep CNN models for pulmonary nodule classification: model modification, model integration, and transfer learning. *Journal of X-Ray Science and Technology*.

[16] Mansouri M., Aran S., Shaqdan K. W., Abujudeh H. H. (2016). Rating and classification of incident reporting in radiology in a large academic medical center. *Current Problems in Diagnostic Radiology*.

[17] Wang S., Wang R., Zhang S. (2018). 3D convolutional neural network for differentiating pre-invasive lesions from invasive adenocarcinomas appearing as ground-glass nodules with diameters ≤3 cm using HRCT. *Quantitative Imaging in Medicine and Surgery*.

[18] Reddy U. J., Reddy B. R. V. R., Reddy B. E. (2019). Recognition of lung cancer using machine learning mechanisms with fuzzy neural networks. *Traitement Du Signal*.

[19] Kang G., Liu K., Hou B., Zhang N. (2017). 3D multi-view convolutional neural networks for lung nodule classification. *PLoS One*.

[20] Lei Y., Tian Y., Shan H., Zhang J., Wang G., Kalra M. K. (2019). Shape and margin-aware lung nodule classification in low-dose CT images via soft activation mapping. *Medical Image Analysis*.

[21] Shan H., Wang G., Kalra M. K., De Souza R. C., Zhang J. Enhancing transferability of features from pretrained deep neural networks for lung nodule classification.

[22] Weston J., Lin C.-J. (2007). Scaling learning algorithms towards AI. *Large-Scale Kernel Machines*.

[23] Satti P., Sharma N., Garg B. (2020). Min-max average pooling based filter for impulse noise removal. *IEEE Signal Processing Letters*.

[24] Moon J., Kim H., Lee B. (2018). View-point invariant 3D classification for mobile robots using a convolutional neural network. *International Journal of Control, Automation and Systems*.

[25] Xie Y., Dai W., Hu Z., Liu Y., Li C., Pu X. (2019). A novel convolutional neural network architecture for SAR target recognition. *Journal of Sensors*.

[26] Winkels M., Cohen T. S. (2019). Pulmonary nodule detection in CT scans with equivariant CNNs. *Medical Image Analysis*.

[27] Neelapu R., Lavanya Devi G., Srinivasa Rao K. (2018). Deep learning based conventional neural network architecture for medical image classification. *Traitement Du Signal*.

[28] Selvaraju R. R., Cogswell M., Das A., Vedantam R., Parikh D., Batra D. Grad-CAM: visual explanations from deep networks via gradient-based localization.

[29] LUNA-16. database available https://luna16.grand-challenge.org/Data/, accessed on 18 December 2019

